# Anti-Inflammatory and Anti-Colon Cancer Activities of Mung Bean Grown in Burkina Faso

**DOI:** 10.1155/2022/7873572

**Published:** 2022-08-09

**Authors:** Wendmintiri Jeanne d'Arc Kabré, Durand Dah-Nouvlessounon, Fatoumata/Ba Hama, N. Arnaud Kohonou, Haziz Sina, Maximin Senou, Lamine Baba-Moussa, Aly Savadogo

**Affiliations:** ^1^Laboratory of Applied Biochemistry and Immunology, Department of Biochemistry and Microbiology, Joseph Ki-Zerbo University, 03 BP 7021, Ouagadougou, Burkina Faso; ^2^Laboratory of Biology and Molecular Typing in Microbiology, Department of Biochemistry and Cell Biology, Faculty of Science and Technology, University of Abomey-Calavi, 05 BP 1604, Cotonou, Benin; ^3^Department of Food Technologies, Institute of Research in Applied Sciences and Technologies (IRSAT), National Center for Scientific and Technical Research, 03 BP 7047, Ouagadougou 03, Burkina Faso; ^4^Experimental and Clinical Biology Laboratory, National School of Applied Biosciences and Biotechnologies, National University of Science, Technology, Engineering and Mathematics (UNSTIM), Dassa-Zoumé, Benin

## Abstract

Widely used in traditional medicine in Asia and recently introduced in Burkina Faso under the name *Beng-tigré*, mung bean is a legume consumed throughout the world and more so in India. The objective of this study was to evaluate the cytotoxicity of the mung bean grown and consumed in Burkina Faso and to study its biological properties such as anti-inflammatory and anticancer activity of the natural and sprouted seeds. The cytotoxicity of the extracts was tested on *Artemia salina* larvae, and the anti-inflammatory activity was evaluated *in vitro* by albumin denaturation method using diclofenac as reference molecule. The anticancer activity of hydro-ethanol extracts was evaluated on rats made cancerous with 1,2-dimethylhydrazine (DMH) using 5-fluorouracil as reference molecule. The results showed that the highest yield of the plant extraction was observed with the hydro-ethanol solvent, both for the natural form of mung bean (MBN) and for its sprouted form (MBG). The cytotoxicity test showed no toxicity of the extracts toward shrimp larvae. The ethanolic extract of germinated mung bean seeds gave the highest anti-inflammatory activity at 95.13 ± 0.22% inhibition with significant difference (*p* < 0.05) between the extracts. Cancer induction with DMH was inhibited by both MBN and MBG extracts. The test of preventive effects of the extracts showed the best activity with significant difference in biochemical results. These results confirm that the mung bean grown in Burkina Faso, as a nontoxic legume, is a functional food that can be integrated into the population's dietary habits for a double interest. Moreover, they open perspectives for the research of active principles of plant origin with anti-inflammatory and anticancer properties.

## 1. Introduction

Nowadays, medicinal plants and natural products from plant biodiversity with pharmacological models have been well studied in several countries as alternative therapies for the treatment of various diseases [1, 2]. A significant number of presently used antimalarial, antioxidant, anthelminthic, anti-inflammatory, and antitumor agents are molecules identified and isolated from plants or functional food plant extracts [3]. In recent years, unhealthy eating habits and diet structure have led to an upward trend in the incidence rate of colon cancer [4].

The gastrointestinal tract is the main site for food digestion and nutrition absorption, and it is the organ that forms the protective barriers [5]. Cancer is the second leading cause of death in the world and remains one of the most worrying diseases today with about 10 million deaths per year, or one in six deaths [6]. Born from the transformation of normal cells into tumor cells, cancer is a multistep process with a precancerous lesion as a starting point. This rapid multiplication of abnormal, unusually growing cells that can invade parts of the body and then migrate to other organs has several causes including poor nutrition. Many studies have shown that the choice of foods consumed over a lifetime can alter the likelihood of carcinogenesis at each stage of the cancer process in a way that reduces risk [7]. In addition, many epidemiological studies have shown that the consumption of food high in phenolic compounds is associated with the prevention of many pathological disorders, including cancer [8]. Currently, there is increasing interest in the consumption of food legumes, not only in the development of new functional ingredients for food enrichment, but also in increasing health and healing potential [9, 10]. Mung bean, the seeds of *Vigna radiata*, is a Fabaceae plant species that is well known as green gram [11]. The seeds are popular food legumes in China, India, Korea, Japan, and other parts of Southeast Asian countries. It is well known for its detoxification activities, recuperation of mentality, ability to alleviate heat stroke, and regulation of a gastrointestinal upset [12]. Widely used in traditional medicine in Asia, mung bean is a legume consumed worldwide and more so in India [13]. Several studies have shown phytochemical profile of mung bean. Twelve phenolic compounds, namely, catechin, epicatechin, p-coumaric acid, ferulic acid, syringic acid, p-hydroxy benzoic acid, protocatechuic acid, gallic acid, vitexin, isovitexin, sinapic acid, and quercetin, have been identified from mung bean [14, 15]. Some phenolic compounds present in this legume, which increase with processes such as germination and fermentation according to [16], could be used in chemoprevention of certain diseases. These compounds are functional food ingredients in mung bean, having a wide range of biological activities including antioxidant [17], anti-inflammatory, antidiabetic [18], antiviral, anticancer, antitumor [13], hepatoprotective [19], antibacterial, antifungal, and other detoxification activities [20]. Thus, the mung bean selected, cultivated, and consumed in Burkina Faso could serve as a functional food in the prevention and management of cancer, the prevalence of which is constantly increasing in the country like in other middle-income countries. The objective of this study was to evaluate the anti-inflammatory capacity and toxicity of different extracts of the mung bean grown in Burkina Faso, in addition to exploring their impact on DMH-induced colon cancer cell proliferation.

## 2. Materials and Methods

### 2.1. Chemicals

The extraction solvents, phosphate buﬀered saline (PBS), were obtained from Sigma-Aldrich Chemical Company (St. Louis, USA). 1,2-Dimethylhydrazine (DMH) was purchased from Macklin (Shanghai Macklin Biochemical Co., Ltd., China). 5-Fluorouracil was purchased from Sigma-Aldrich (St Louis, MO, USA). Biochemical analysis kits were BIOLABO diagnostic kits. All the chemicals and reagents were of analytical grade.

### 2.2. Plant Material and Sample Preparation

The plant material used consists of seeds of mung bean (*Vigna radiata*) obtained from the Belwet structure located in district 2 of the municipality of Ouagadougou, the main promoter of mung bean in Burkina Faso. The mung bean was used in two forms as raw material. These are the natural form (MBN) and the germinated form (MBG). The natural mung bean sample (MBN) was obtained by washing the natural mung bean seeds with demineralized water and then drying them at 60°C for 12 hours. The sprouted mung bean (MBG) sample was obtained by hydrating the natural mung bean seeds with demineralized water for 12 hours before germinating them between two bedded fabrics for 48 hours. After drying at 60°C for 12 hours, the rootlets were removed. A stainless steel grinder (IKA Bro-03-PATACE-018) was used to grind the different samples.

### 2.3. Animal Material and Acclimatization Conditions

The animals used were Wistar rats of EOPS (Exempt from Specific Pathogenic Organisms) health status, aged approximately eight weeks and weighing between 150 g and 200 g. The animals were housed in polypropylene cages integrated with water pots and under hygienic conditions with standard rat food and free access to water. After two weeks of acclimatization at a constant temperature of 22 ± 2°C under a 12/12 h light/dark cycle, the rats were divided into batches for the different tests. The body weight of the rats was recorded at the beginning and at the end of the experiment. This research protocol has been approved by the Scientific Ethics Committee of the Doctoral School (Life Sciences) of the Faculty of Science and Technology (FAST) at the University of Abomey-Calavi (UAC), Benin (No. UAC/FAST/EDSV/1357006).

### 2.4. Preparation of Extracts

For each sample, three types of extracts were made with polar solvents. These were ethanol, water-ethanol mixture (30 : 70, v/v), and methanol. The extraction method described by [21] was used. Briefly, 50 g of sample powder (MBN, MBG) was macerated for 72 h under continuous stirring in 500 mL of each solvent. The macerates were then filtered 3 times with cotton wool and once with Whatman paper. The filtrates obtained were then dried at 40°C in the oven until complete evaporation. The residues obtained after drying constituted the extracts derived from each solvent and were used for the study of different biological activities. The yield of the crude extract of each solvent was determined by the ratio of the mass of the dry extract obtained to the mass of the treated plant material.

### 2.5. Evaluation of Anti-Inflammatory Activity of Extracts

The *in vitro* anti-inflammatory activity of the different extracts of MBN and MBG was evaluated following an adaptation of the protocol described by [22]. The reaction mixture (250 *µ*L) consisted of 10 *µ*L of egg albumin, 140 *µ*L of phosphate buffered saline (PBS, pH 6.4), and 100 *µ*L of extract of concentration 100 mg/mL. A series of 10 successive dilutions of each extract was made from 100 mg/mL sample solution dissolved in methanol or distilled water. The mixtures were incubated in the dark for 15 min and then heated at 70°C for 5 min. Absorbance was measured at 660 nm after cooling against a blank prepared under the same conditions using Thermo Fisher Scientific BioMate 3S Spectrophotometer, USA.

(1) $$\begin{array}{c} \%\text{ Inh }=\frac{\text{Abs Control}-\text{Abs Sample}}{\text{Abs Control}}, \end{array}$$

where % Inh is the inhibition percentage, Abs Control is the absorbance of control, and Abs Sample is the absorbance of sample.

### 2.6. Evaluation of Anticancer Activity

It was performed *in vivo* with the Wistar rats following the protocol adapted from [23]. All the handling procedures also considered the guidelines for animal models of cancer study. The effects of mung bean extracts on anarchic proliferation of the rat's colon cells were tested by assay of biochemical parameters and histopathological observations. 1,2-Dimethylhydrazine (DMH) was the molecule used to induce colon cancer *in vivo*. It was prepared in 1 Mm EDTA saline pH 7.1 for subcutaneous injection at 45 mg/kg body weight. The reference molecule used was 5-fluorouracil at 0.6 mL/kg/body weight. The extracts were administered by gavage at 300 mg/mL with a volume of 100 ml/kg body weight.

### 2.7. Experimental Design

Rats were randomly assorted and bodily marked for indication. A number of 36 rats were divided into 9 groups of 4 rats each according to their body weight. All animals were provided with food and water ad libitum throughout the experimental period.

  Group 1: negative control. These rats received plain water and food during the six weeks of the experiment.
  Group 2: positive control, DMH-treated. These rats received twice a week a subcutaneous injection of DMH during the six weeks of the experiment.
  Group 3: inhibition effect of extracts. These rats received a subcutaneous injection of DMH twice a week and MBN extract (300 mg/kg) daily.
  Group 4: inhibition effect of extracts. These rats received a subcutaneous injection of DMH twice a week and MBG extract (300 mg/kg) daily.
  Group 5: curative effect of extracts. These rats received a subcutaneous injection of DMH twice a week for six weeks; at the third week, MBN extract (300 mg/kg) was applied daily until the end of the six weeks.
  Group 6: curative effect of extracts. These rats received a subcutaneous injection of DMH twice a week for six weeks; at the third week, MBG extract (300 mg/kg) was applied daily until the end of the six weeks.
  Group 7: preventive effect of extracts. These rats received MBN extracts (300 mg/kg) daily throughout the six weeks. At the third week, a subcutaneous injection of DMH was applied twice a week until the end of the six weeks.
  Group 8: preventive effect of extracts. These rats received MBG extracts (300 mg/kg) daily throughout the six weeks. At the third week, a subcutaneous injection of DMH was applied twice a week until the end of the six weeks.
  Group 9: effects of the reference molecule. These rats received a subcutaneous injection of DMH twice a week combined with an intravenous injection of 5-fluorouracil (0.6 mL/kg).

### 2.8. Determination of Biochemical Parameters

In addition to the weight of the animals, biochemical parameters were measured before and at the end of the experiment in order to assess the biochemical changes that might occur during the experiment. Blood sampling was performed by puncturing the retro-orbital sinus of animals (under diethyl ether anesthesia). Hematocrit, hemoglobin, red cell count, white blood cell count, leukocyte, and neutrophils were measured with animal total blood samples. Besides, the blood was centrifuged at 3000 rpm and the plasma collected and analyzed with BIOLABO (FRANCE) diagnostic kits. Following the manufacturer's instructions, the plasma concentrations of creatinine (kit REF 80107, LOT 012042A) and urea (kit REF 92032, LOT 041915A), as well as aspartate aminotransferase (AST) and alanine aminotransferase (ALT) activities (kit REF 51830, LOT 072105A7), were determined.

### 2.9. Anatomical Observations

After six weeks of follow-up, all the animals were sacrificed under the same fasting conditions at night (10 p.m.) under yellow light according to the protocol of [23]. Liver, kidneys, and colon were removed and rinsed with saline. The colon was opened longitudinally and examined microscopically to observe the presence of multiple identifiable lesions and the appearance of aberrant crypt foci. The colon segments containing the multiple plaque lesions (MPL) were dissected, fixed immediately in 10% formalin over paraffin, sectioned, and stained with hematoxylin and eosin for histopathological observations. The liver and kidneys were then placed in 10% formalin for histological sections.

### 2.10. Evaluation of the Cytotoxicity of Mung Bean Extracts

The cytotoxic effect of the extracts was evaluated following an adaptation of the method described by [24]. Larvae were obtained by hatching 10 mg of freeze-dried *Artemia* eggs under continuous agitation in 1L of seawater for 72 h. The number of surviving larvae in the different concentrations of extract was counted after 24 h of incubation. For each extract, the lethal concentration (LC_50_) was determined from the regression line obtained from the curve representing the number of surviving larvae as a function of the extract concentration.

### 2.11. Statistical Analysis

Microsoft Excel 2016 spreadsheet was used for data processing. GraphPad Prism 8 software was used for the analyses of variances. The differences were considered significant at *p* < 0.05.

## 3. Results and Discussion

### 3.1. Results

#### 3.1.1. Extract Yield

The yield of the different extracts expressed as a percentage of the sample powder mass is summarized in Table 1. The table shows a wide variation in yield depending on the extraction solvent used. MBG extracts gave higher yield than MBN extracts. The hydro-ethanol extract gives the best yield for both MBN and MBG.

#### 3.1.2. Anti-Inflammatory Activities

The anti-inflammatory activity of the tested extracts is summarized in Table 2. The effect of the extracts on albumin denaturation expressed here by the rate of inhibition varies according to the mung bean sample (MBG and MBN) and extract types. The hydro-ethanolic and methanolic extracts of MBG showed no effect on the denaturation of the protein used (albumin). Besides, the ethanolic extract of MBG has shown a high inhibition rate (95.13 ± 0.22%) of albumin denaturation. Furthermore, the results show the good activity of MBN extracts. Indeed, for MBN, the ethanolic extract recorded the highest inhibition rate (93.14 ± 0.36%) of albumin denaturation while methanolic extract showed the lowest one (28.72 ± 0.35%). Moreover, for the two forms of mung bean (MBN and MBG), although the ethanolic extract of MBG showed higher percentage of inhibition, the ethanolic extract of MBN had lower inhibitory concentration (IC_50_ < 12.5 mg/mL).

### 3.2. Anticancer Activity

#### 3.2.1. Macroscopic Analysis of Colon

For macroscopic observation, the longitudinally opened colons were carefully examined for the presence of nodular lesions on the surface of the colonic mucosa. Indeed, comparison of the colonic surface of rats in group R1 (without DMH or extract) and rats in group R2 (treated with DMH) showed the presence of visible tumors in the DMH-treated rats (R2). These visible tumors were considered to be the early centers of tumorigenesis; thus, DMH at 45 mg/kg actually induced colon cancer. In addition, there was a large difference between the colonic surface area of rats in the R2 group (treated with DMH) and those of rats in the R3 group (MBN + DMH in inhibitory treatment), R4 (MBG + DMH in inhibitory treatment), R5 (MBN + DMH curative treatment), R6 (MBG + DMH curative treatment), R7 (MBN + DMH preventive treatment), R8 (MBG + DMH preventive treatment), and R9 (5-fluorouracil treatment).

#### 3.2.2. Biochemical Analyses

The variation of biochemical parameters is presented in Table 3. All biochemical parameters of the rats showed highly significant variations (*p* < 0.05) compared to the control. According to the parameters, the DMH-treated rats (R2) showed clearly different mean values (*p* < 0.05). For the parameters measured with the animal's total blood samples (hematocrits, hemoglobin, number of red blood cells, number of white blood cells, leucocytes, and neutrophils), among the different treatments carried out, a variation was observed with two parameters (red blood cells and white blood cells) for the evaluation of the inhibition effect (R3 and R4). Indeed, in group R3 (MBN+ DMH) there is an increase (2.93 ± 0.27 to 4.31 ± 0.06) in the number of white blood cells and neutrophils (27.5 ± 1.5 to 41.00 ± 1.00). In contrast, there was a decrease (5.28 ± 0.32 to 2.24 ± 0.13) in the number of red blood cells in group R4 (MBG+ DMH). Apart from these two parameters, whose difference may also be related to bacterial infection, no variation (*p* > 0.05) was observed for all other parameters in relation to preventive, curative, and reference treatments (5-fluorouracil). These observations suggest that MBN and MBG extracts neutralize the effect of DMH on blood parameters. These extracts have an effect comparable to that of 5-fluorouracil used as a reference molecule, which demonstrates their effectiveness with regard to blood parameters.

For the plasma concentration of creatinine, urea, aspartate aminotransferase (AST), and alanine aminotransferase (ALT), a change in the plasma concentrations of AST, ALT, and creatinine was observed in groups R3 and R4 with inhibition treatment. However, the change is reversed when switching from MBN extract to MBG extract. These observations show that MBG extract inhibits the effects of DMH on plasma parameters better than MBN extract. Furthermore, between the preventive treatment and the 5-fluorouracil treatment, the plasma parameters do not show any variation except with AST (86.5 ± 2.5 to 109.5 ± 0.5) for MBN extract. In general, the preventive treatment showed better efficacy of the extracts considering the biochemical parameters.

### 3.3. Histological Analysis

#### 3.3.1. Observation of the Colon

The effects of DMH and the different treatments on the rat colon are shown in Figure 1. In the DMH-treated group (R2), the colonic mucosa shows atypia in places. The glandular epithelium is unrecognizable and resembles a Lieberkühnian adenocarcinoma. The glands (G) are recognizable in places. These observations show that DMH induced uncontrolled cell proliferation in the rat colon.

In the groups of rats that received inhibition treatment (groups R3 and R4 treated with MBN + DMH and MBG + DMH, respectively), the colonic mucosa does not show atypia. The unstratified lining epithelium (ER) is characteristic with its simple columnar cells with microvilli (absorptive epithelium). Lieberkühn's glands (G) are typical. These observations show that both extracts (MBN and MBG) inhibited the action of DMH on the colon of treated rats by preventing uncontrolled cell proliferation compared to the positive control (DMH-treated).

Considering the curative treatment groups (groups R5 and R6 treated with MBG + DMH and MBN + DMH, respectively), some foci of atypia remained. In group R5 (treated with MBG + DMH), there are more recognizable glands than in the control group treated with DMH (R2). In group R6 (treated with MBN + DMH), the lining epithelium shows some foci of cell proliferation (PC). Lieberkühn's glands (G) are more typical in group R5 (treated with MBN + DMH). These observations show that curative treatment is less effective. However, MBG extract showed better curative activity than MBN extract.

In the preventive treatment groups (groups R7 and R8 treated with MBN + DMH and MBG + DMH, respectively) and in the group treated with 5-fluorouracil (R9), the colonic mucosa did not show atypia. Absorbent lining epithelium (ER) and Lieberkühn's glands (G) were characteristic. For the preventive treatment, MBN and MBG extracts show similar effects to the reference molecule, showing a strong preventive activity of both extracts. The preventive treatment is therefore more effective than the curative treatment.

#### 3.3.2. Observation of the Liver

Besides the observations on the colon, the possible effects of DMH on the liver were examined.  Figure 2 shows the histology of the liver of experimental Wistar rats. The liver parenchyma showed no visible atypia in the different groups (DMH, MBN, MBG, and 5-fluorouracil). The hepatocytes (H) are well organized in cords around the centrilobular veins (CV). The venous sinusoids (S) are clearly visible between the hepatocyte cords. These observations show that DMH did not have a harmful effect on the liver of treated rats.

#### 3.3.3. Observation of the Kidneys

Figure 3 shows the histopathology of the kidneys of the experimental rats. In the DMH-treated group (positive control group), the renal parenchyma shows cellular debris (arrows) in some tubular lumens, indicating cellular damage. In the other groups (treated with MBN, MBG, and 5-fluorouracil), the appearance of the parenchyma is typical with characteristic glomeruli (G) and renal tubules (TR). The tubular lumens are clearly visible. These observations show that only DMH had a moderate negative effect on the kidneys of treated rats.

#### 3.3.4. Cytotoxicity of Extracts

The cytotoxicity of MBN and MBG extracts tested on *Artemia salina* larvae is presented in Figure 4. Mung bean, whether natural or sprouted, showed no toxicity or lethal dose in larvae. The ethanolic extract of MBG recorded more larval loss at high concentrations, followed by its methanolic extract.

## 4. Discussion

The extraction yield showed that hydro-ethanolic extracts had a better yield compared to ethanolic and methanolic extracts. The percentage of extracts always higher for MBG than for MBN regardless of the solvent used allows us to conclude that MBG has more bioactive molecules than MBN. Our results are in agreement with those of [25] who reported that the extraction yield increased with germination. Germination is then a process that leads to physicochemical changes and biochemical modifications that can increase the content of some biomolecules.

The mung bean grown in Burkina Faso showed no toxicity with reference to the toxicity scale established by [26]. All the extracts from both MBN and MBG had LD_50_ > 0.1 mg/mL. Mung bean, whether plain or sprouted, is a healthy food for both children and adults and is not contraindicated for the sick.

Our results also show good anti-inflammatory activity of both MBN and MBG. Several experimental studies have well established the modulation of inflammatory effects by mung bean [27]. In this study, MBN ethanolic extracts and MBG hydro-ethanolic extracts have good inhibition of protein denaturation compared to the reference molecule (diclofenac sodium) with the lower IC_50_ < 12.5 mg/mL. Reference [28] reported that the aqueous extract of mung bean husk is protective against sepsis. Moreover, [29] noted that sprouted mung bean had a protective effect on arthritis which can be attributed to a combination of anti-inflammatory and antioxidant effects capable of acting on various pharmacological targets.

Our results showed that the subcutaneous injection of DMH-induced tumors in the colons of the rats that received it, as evidenced by the colons of the R2 group rats (DMH-treated). DMH would then be an effective molecule in the induction of cancer in rats in a short time. This observation on DMH was made by Sharma et al. [23] who also reported the efficacy of DMH in cancer induction in experimental animal models. For the macroscopic analysis, the absence of visible tumor in the colons of groups R3, 4, 5, 6, 7, 8, and 9 in comparison to those of group R2 attests that the extracts of both MBN and MBG, as well as the reference molecule, had an effect on DMH-induced cell proliferation. Lee et al. [30] as well as Singh et al. [31] reported the presence of flavonoids and tannins in the cotyledons and integuments of mung bean. The work of Stavric and Matula [32] concluded that these polyphenols possess antitumor and anticarcinogenic properties. We can therefore conclude that these flavonoids and tannins are present in our extracts and have contributed to the inhibition of the carcinogenic effects of DMH. Moreover, the aspects of the colon of the rats given the MBG extracts are even closer to those of the R1 group (negative control group) than to those given the MBN. The germination process increased the content of some biomolecules in mung bean, which may contribute to the inhibition of DMH effects. References [16, 33] found that phenolic acid content increases with seed germination.

The results of biochemical parameters like hematocrit, hemoglobin, uremia, aspartate aminotransferase (AST), alanine aminotransferase (ALT), and creatinine showed disparity between different groups of rats, mainly between the rats of group R2 and the rest of the rats of other groups. All the biochemical parameters of group R2 rats showed a decrease or an increase with a significant difference (*p* < 0.05) between the beginning and the end of the experiment. Indeed, the rats of group R2 showed a significant decrease in hematocrit and hemoglobin level unlike those of the rats of the other groups which also showed a decrease but it was not significant. The decrease in hematocrit level with a significant difference in group R2 rats reflects anemia in these rats due to probable inflammation caused by DMH; this is evidenced by the decrease in their hemoglobin levels. The increase in AST and ALT transaminase levels in some cases, with a highly significant difference (*p* < 0.0001) in R2 group rats, reflects DMH-induced liver damage, the effect of which was attenuated in rats fed with the different MBN and MBG extracts. Liver biomarkers such as alanine aminotransferase (ALT) and aspartate aminotransferase (AST) are generally used for clinical diagnosis and estimation of disorders involving functional liver impairment or morphological liver damage [34]. The results of biochemical tests show that MBN and MBG extracts attenuated significant variations in the activity of these enzymes compared to R2 group. Reference [35] found a decrease in AST and ALT levels in hepatocyte mice after 14 days of consumption of aqueous mung bean extracts. All these biochemical results show a metabolic disorder, which is even more pronounced in R2 group rats, as evidenced by their urea levels which increased very significantly. Indeed, as in the macroscopic observation and biochemical tests, the 5-fluorouracil used in our study as a reference molecule also showed its efficacy with the histological analyses. 5-Fluorouracil (5-FU) is the first choice chemotherapeutic agent in the treatment of colorectal cancer patients [36]. Intracellular metabolites of 5-FU can exert cytotoxic effects via inhibition of thymidylate synthetase, or incorporation into RNA and DNA, events that ultimately activate apoptosis [37]. Increasing the dose of systemically administered 5-FU would generate unacceptable levels of toxicity to normal cells, particularly those in the bone marrow and gastrointestinal tract, leading to severe adverse effects [36]. Histological analysis showed no cell damage due to 5-fluorouracil, reflecting the correct dose used in our study. All these observations were confirmed and better appreciated by histological analysis. Reference [25] reported antiproliferative effects of mung bean extracts germinated for 48 hours, tested on different drug-resistant colon cancer cell lines, T84 and HCT-18, as well as on a non-tumorous CCD-18 line. Similarly, [38] showed that bioactive components of mung bean seeds have a wide range of activities such as anticancer, antihyperlipidemic, and antihypertensive activities. Reference [39] reported an in vivo study suggesting that aqueous extracts of fermented mung bean could delay the formation of breast cancer and reduce the mitotic division of the tumor by stimulating the cytokine production of T cells. These observations indicate that consumption of mung beans grown in Burkina Faso may reduce the risk of digestive tract cancer. Epidemiological studies have also suggested that bean consumption reduces the prevalence of cancers, including colon, breast, prostate, and adenocarcinoma [40]. Other studies have reported that eating beans more than twice a week was associated with a marked reduction (47%) in the risk of colon cancer [41] and prostate cancer [40]. Reference [42] reported that regular consumption of beans in rats was found to decrease the morphology of azomethane-induced tumors by up to 50%.

## 5. Conclusion

The present study evaluated the anti-inflammatory and anticancer activities of organic extracts of mung bean grown in Burkina Faso. The data obtained revealed that the mung bean grown in Burkina Faso has pharmacological properties that may have beneficial effects on the health of consumers. The cytotoxicity study showed that the extracts were not toxic at the dose studied (20 mg/ml). MBN and MBG have good anti-inflammatory activity which can help relieve sepsis in frail people and arthritis in elderly subjects. In addition, mung bean grown in Burkina Faso has shown good anticancer activity. In cancer-prone Wistar rats, MBG was found to be more effective than MBN in preventing and curing cancer by inhibiting DMH-induced cancer cell proliferation. While the choice of certain foods in the diet may be at the root of the progressive onset of some degenerative diseases, other food choices could contribute to their prevention and alleviation. The mung bean grown in Burkina Faso is a functional food that can contribute to the management of degenerative diseases. These results open up prospects for the search for active principles of plant origin with anti-inflammatory and anticancer properties and may constitute an answer contributing to the prevention of degenerative diseases.

## Figures and Tables

**Figure 1:** Histology of the colon of experimental Wistar rats (original magnification ×400). R2: DMH treatment; R3: inhibition effect of MBN extracts; R4: inhibition effect of MBG extracts; R5: curative effect of MBG extracts; R6: curative effect of MBN extracts; R7: preventive effect of MBN extracts; R8: preventive effect of MBG extracts; R9: effects of 5-fluorouracil used as reference molecule; G: Lieberkühn's glands; ER: lining epithelium; PC: foci of cell proliferation.

**Figure 2:** Histology of the liver of experimental Wistar rats (original magnification ×400). R2: DMH treatment; R3: inhibition effect of MBN extracts; R4: inhibition effect of MBG extracts; R5: curative effect of MBN extracts; R6: curative effect of MBG extracts; R7: preventive effect of MBN extracts; R8: preventive effect of MBG extracts; R9: effects of 5-fluorouracil used as reference molecule; VC: centrilobular veins; H: hepatocytes; S: sinusoids.

**Figure 3:** Histology of the kidneys of experimental Wistar rats (original magnification ×400). R2: DMH treatment; R3: inhibition effect of MBN extracts; R4: inhibition effect of MBG extracts; R5: curative effect of MBN extracts; R6: curative effect of MBG extracts; R7: preventive effect of MBN extracts; R8: preventive effect of MBG extracts; R9: effects of 5-fluorouracil used as reference molecule; TR: renal tubules; G: glomeruli.

**Figure 4:** Representation of the number of surviving larvae as a function of extract concentration.

**Table 1:** Plant material extraction yield.

Extracts	Yields (%)	
	Natural mung bean (MBN)	Germinated mung bean (MBG)
Ethanolic	1.42	1.66
Hydro-ethanolic	4.66	8.72
Methanolic	1.27	2.12

**Table 2:** Anti-inflammatory activity and IC_50_ of extracts.

	Extracts	Inhibition rate (%)	IC_50_ (mg/mL)
MBN	Ethanolic	93.14 ± 0.36	<12.5
	Hydro-ethanolic	81.31 ± 0.78	43 ± 0.28
	Methanolic	28.72 ± 0.35	>100

MBG	Ethanolic	95.13 ± 0.22	20.5 ± 0.46
	Hydro-ethanolic	nd	—
	Methanolic	nd	—

MBN: natural mung bean, MBG: germinated mung bean.

**Table 3:** Variation of biochemical parameters observed in rats of different batches (mean ± standard deviation).

Parameters	R1	R2	R3	R4	R5	R6	R7	R8	R9
Htei	37.5a ± 0.5	38.5a ± 0.5	36.5a ± 0.5	34.5a ± 0.5	35.5a ± 0.5	36.00a ± 0.00	34.5a ± 0.5	33.5a ± 0.5	36.5a ± 0.5
Htef	37.5a ± 0.5	19.5b ± 0.5	36.00a ± 0.00	35.5a ± 0.5	37.00a ± 0.00	37.5a ± 0.5	35.00a ± 0.00	34.5a ± 0.5	36.5a ± 0.5
HBi	12.15a ± 0.15	12.85a ± 0.15	10.77a ± 0.55	9.5a ± 0.50	11.31a ± 0.15	10.15a ± 1.14	10.34a ± 0.12	9.45a ± 0.22	11.47a ± 0.14
HBf	11.10b ± 0.10	3.50b ± 0.5	11.32a ± 0.05	10.67a ± 0.47	11.73a ± 0.19	9.5a ± 0.5	11.45a ± 0.13	9.94a ± 0.31	11.44a ± 0.07
GRi	4.12a ± 0.06	4.12a ± 0.15	3.21a ± 0.55	5.28a ± 0.32	5.42a ± 0.21	5.23a ± 0.00	3.87a ± 0.11	4.68a ± 0.46	4.45a ± 0.16
GRf	4.11a ± 0.01	1.16b ± 0.06	3.41a ± 0.02	2.24b ± 0.13	4.45a ± 0.22	4.01a ± 0.00	4.12a ± 0.01	3.65a ± 1.02	4.07a ± 0.06
GBi	5.22a ± 0.10	6.00a ± 0.39	2.93b ± 0.27	3.44a ± 0.48	4.26a ± 0.03	6.28a ± 0.95	3.45a ± 0.22	4.67a ± 0.49	4.16a ± 0.03
GBf	3.54b ± 0.11	1.77b ± 0.54	4.31a ± 0.06	5.83a ± 0.40	3.89a ± 0.37	5.02a ± 0.09	3.48a ± 0.34	4.29a ± 0.17	4.26a ± 0.07
Li	23.5a ± 4.5	20.5b ± 0.5	17.00a ± 1.00	17.00a ± 1.00	18.00a ± 0.00	17.00a ± 0.00	23.5a ± 1.5	18.00a ± 2.00	19.5a ± 0.5
Lf	21.5a ± 1.5	43.00a ± 4	20.5a ±.05	20.00a ± 0.00	17.5a ± 1.5	21.5a ± 0.5	24.5a ± 1.5	20.5a ± 1.5	19.5a ± 0.5
Ni	40.00a ± 0.00	40.5b ± 1.5	27.5b ± 1.5	42.00a ± 3.00	64.00a ± 1.00	33.00a ± 4.00	34.00a ± 5.00	40.5a ± 1.5	41.5a ± 0.5
Nf	40.00a ± 0.00	87.5a ± 5.5	41.00a ± 1.00	56.5a ± 28.5	66.00a ± 1.00	54.5a ± 5.5	40.5a ± 0.5	39.5a ± 0.5	42.00a ± 0.00
Ureai	0.42a ± 0.01	0.33b ± 0.04	0.19a ± 0.03	0.19a ± 0.01	0.14a ± 0.01	0.19a ± 0.04	0.55a ± 0.42	0.36a ± 0.17	0.38a ± 0.02
Ureaf	0.39a ± 0.03	3.87a ± 0.11	0.20a ± 0.04	0.25a ± 0.08	0.38a ± 0.19	1.16a ± 0.04	0.21a ± 0.02	0.16a ± 0.01	0.41a ± 0.00
ASTi	96a ± 4	100.00b ± 2	120.5a ± 12	117.5a ± 6.5	118.5a ± 0.5	103.00b ± 1.00	86.5b ± 2.5	163.00a ± 1.00	104.5a ± 1.5
ASTf	105a ± 1	356.00a ± 47	122.5a ± 0.5	97.00b ± 1.00	87.00b ± 9.00	129.00a ± 3.00	109.5a ± 0.5	128.00b ± 3.5	107.00a ± 2.00
ALTi	101a ± 1	81.00b ± 17	92.5a ± 3.5	88.00b ± 2.00	120.5a ± 2.5	125.5a ± 2.5	116.00a ± 2.00	127.00a ± 5.00	106.00a ± 2.00
ALTf	96a ± 2	256.00a ± 8	75.5a ± 13.5	98.5a ± 0.5	113.00a ± 11.00	113.00b ± 1.00	115.00a ± 19.00	107.5b ± 4.5	101.5a ± 1.5
Creati	7.55a ± 0.35	9.47b ± 0.23	7.38a ± 0.42	7.24a ± 0.9	11.31a ± 3.91	8.21a ± 0.12	7.1a ± 0.2	8.75a ± 0.15	7.17a ± 0.07
Creatf	8.40a ± 0.20	15.23a ± 1.9	8.43a ± 0.81	6.38a ± 0.7	5.25b ± 0.65	10.68a ± 0.55	7.7a ± 0.5	9.80a ± 2.20	7.15a ± 0.03

R1: negative control; R2: DMH treatment; R3: inhibition effect of MBN extracts; R4: inhibition effect of MBG extracts; R5: curative effect of MBN extracts; R6: curative effect of MBG extracts; R7: preventive effect of MBN extracts; R8: preventive effect of MBG extracts; R9: effects of 5-fluorouracil used as reference molecule. Intra-column means followed by the different letters differ significantly at the 5% level for each constituted batch. Htei: initial hematocrit level; Htef: final hematocrit level; HBi: initial hemoglobin level; HBf: final hemoglobin level; GRi: initial red cell count; GRf: final red cell count; GBi: initial white blood cell count; GBf: final white blood cell count; Li: initial leukocyte; Lf: final leukocyte; Ni: initial neutrophils; Nf: final neutrophils; Ureai: initial uremia; Ureaf: final uremia; ASTi: initial aspartate aminotransferase; ASTf: final aspartate aminotransferase; ALTi: initial alanine aminotransferase; ALTf: final alanine aminotransferase; Creati: initial creatinine; Creatf: final creatinine.

## Data Availability

The data used to support the findings of this study are available from the corresponding author upon request.
